# A Machine Learning Applied Diagnosis Method for Subcutaneous Cyst by Ultrasonography

**DOI:** 10.1155/2022/1526540

**Published:** 2022-10-17

**Authors:** Hao Feng, Qian Tang, Zhengyu Yu, Hua Tang, Ming Yin, An Wei

**Affiliations:** ^1^Department of Dermatology, Hunan Provincial People's Hospital (The First Affiliated Hospital of Hunan Normal University), Changsha 410005, China; ^2^Faculty of Engineering and IT, University of Technology, Sydney, Sydney, NSW 2007, Australia; ^3^Department of Ultrasound, Hunan Provincial People's Hospital (The First Affiliated Hospital of Hunan Normal University), Changsha 410005, China

## Abstract

For decades, ultrasound images have been widely used in the detection of various diseases due to their high security and efficiency. However, reading ultrasound images requires years of experience and training. In order to support the diagnosis of clinicians and reduce the workload of doctors, many ultrasonic computer aided diagnostic systems have been proposed. In recent years, the success of deep learning in image classification and segmentation has made more and more scholars realize the potential performance improvement brought by the application of deep learning in ultrasonic computer-aided diagnosis systems. This study is aimed at applying several machine learning algorithms and develop a machine learning method to diagnose subcutaneous cyst. Clinical features are extracted from datasets and images of ultrasonography of 132 patients from Hunan Provincial People's Hospital in China. All datasets are separated into 70% training and 30% testing. Four kinds of machine learning algorithms including decision tree (DT), support vector machine (SVM), *K*-nearest neighbors (KNN), and neural networks (NN) had been approached to determine the best performance. Compared with all the results from each feature, SVM achieved the best performance from 91.7% to 100%. Results show that SVM performed the highest accuracy in the diagnosis of subcutaneous cyst by ultrasonography, which provide a good reference in further application to clinical practice of ultrasonography of subcutaneous cyst.

## 1. Introduction

Subcutaneous cyst occurs especially at younger age, especially in the head, arms, and back in youth. It is a soft or a plurality of soft or firm balls with diameters ranging from 1 to approximately 3 cm. Subcutaneous cyst is buried in the skin or subcutaneous tissue and adheres to the skin and the base can move. There are small openings on the skin. When the cyst is pushed, it adheres tightly to the skin. Small pit appears when it is slightly depressed, which is the opening of the duct where the gland directly reaches the skin surface. Some openings are stuffed with a black pimple-like plug to squeeze out white wax-like substances [1–3]. The ultrasonic images of superficial epidermoid cyst have certain specificity. The advantages of ultrasound include high spatial resolution, portability, convenience, and low cost. It is important to be able to combine the physical examination results with the patient's medical history in ultrasonic examination. In addition, real-time imaging allows manual compression, limb movement, muscle contraction, and direct interaction with patients during scanning [4]. By summarizing and analyzing its acoustic features, it can effectively improve the correct rate of clinical diagnosis and reduce misdiagnosis and missed diagnosis [5, 6]. However, one disadvantage of ultrasound is when the disease occurs in deeper soft tissues. In these cases, the image resolution is reduced, and auxiliary information about the mass, such as physical examination results and medical history, may be blurred [7].

Machine learning is one of the branch in artificial intelligence and has been widely used in multidisciplinary research fields [8, 9], which is related to computer science, statistics, and information theory [10, 11]. Algorithms are used to analyze data and try to explore potential patterns hidden in data to predict new information in machine learning [8, 12], with high precision, high speed, and convenient expansion [13, 14]. The main application fields of deep learning in ultrasound computer-aided diagnosis system include breast disease diagnosis [15], liver disease diagnosis [16], fetal ultrasound standard plane detection [17], thyroid nodule diagnosis [18], and carotid artery ultrasound image classification [19]. In recent years, machine learning algorithms, such as decision tree (DT), support vector machine (SVM), *K*-nearest neighbors (KNN), and neural networks (NN), have been more and more frequently applied in medical field [20–23].

However, limited relative studies on machine learning in the diagnosis of subcutaneous cyst based on ultrasonography have been reported. Thus, the motivation and novelty of this study were to apply several machine learning algorithms to diagnose subcutaneous cyst from clinical features extracted from datasets and images of ultrasonography and find a powerful alternative method for ultrasonic diagnosis of subcutaneous cysts.

## 2. Materials and Methods

### 2.1. Data Acquisition

All datasets in this article are from Hunan Provincial People's Hospital in China. There are 133 patients that participated. Each patient has five ultrasound images record with 19 clinical features extracted including gender, age, none blood flow, dotted blood flow, dot-bar blood flow, rich blood flow, none echo, mixed echo, low echo, medium echo, high echo, uniform internal echo, nonuniform internal echo, clear boundary, unclear boundary, regular form, irregular form, strong spot, and changes of parenchyma echo.  Figure 1 illustrates sample ultrasound images of subcutaneous cyst.

### 2.2. Data Preparation

A machine learning applied method is proposed to diagnose subcutaneous cyst in this article. Clinical features are extracted from datasets and images of ultrasonography.  Figure 2 displays the workflow processes for the machine learning applied diagnosis method in several steps, which are presented in the following:

1. Extract clinical features from datasets and ultrasound images
2. Allocate feature types: there are two different feature types in our method, categorical and numerical. To improve the accuracy of the diagnosis method, we allocated these features into two types, Table 1 presents all the features and types
3. Training algorithms: machine learning algorithms, such as decision tree (DT), support vector machine (SVM), *K*-nearest neighbors (KNN), and neural networks (NN), had been approached to determine the best performance. The result indicated that the best accurate algorithm is SVM. Feature 1 (gender) and feature 2 (age) are excluded from target features, as they are basic information of the patient, they do not change or are not affected by cysts lesions. Therefore, the target features in this research are 17 features, which are from feature 3 to feature 19. In the training stage, we start from target feature 3, the results indicated that SVM provided the highest accuracy
4. Testing algorithm: in this stage, the rest 30% of the datasets is processed by SVM. We use the same target feature as the previous training. SVM achieves 100% accuracy
5. Testing target features: each target feature is trained and tested to validate the reliability of SVM. The rest target features are from feature 4 to feature 19. We compared with all the results from each feature, SVM still achieved the best performance from 91.7% to 100%. This is a significant accuracy in diagnosing subcutaneous cyst

Statistical Processing

## 3. Results

### 3.1. Training Process

Four different types of machine algorithms are applied. We separated datasets into two parts, 70% for training and 30% for testing. 19 features from 132 patients are computed. Since feature 1 and feature 2 are gender and age, they are general information of patients and will not be affected by any cyst lesions, and the target features in this research are from feature 3 to feature 19. Initially, we set feature 3, none blood flow, as the target feature, and the rest of the features are attributes. To avoid datasets overfitting, we use 5 cross-validation folds. After processing the training by using DT, SVM, KNN, and ANN, the accuracy results are 99.2%, 100%, 92.4%, and 98.5%, respectively. SVM provides best result for the diagnosis method.  Table 2 indicates the accuracy result for the training process.

### 3.2. Testing Process

To validate the reliability of the method, SVM is tested by using the rest 30% of the datasets. The target features are the same as the previous training, which are from feature 3 to feature 19. We start setting the target feature from feature 3. We also use 5 cross validation folds to avoid datasets overfitting. As shown in Table 3, the testing results slightly changed to DT (96.2%), SVM (100%), KNN (95.5%), and ANN (98.5). Comparing with the results, SVM still achieves 100% accuracy. It is the best algorithm for the diagnosis method when we set the target feature as feature 3.

### 3.3. Training and Testing for Each Target Feature

In the previous stage, we trained and tested feature 3 as a target feature, and the result indicated that SVM achieved the best accuracy. Further training and testing are approached for each target feature, from feature 4 to feature 19.  Table 4 indicates the testing results for 17 target features. In Table 4, the target features are trained and tested by using DT, SVM, KNN, and ANN. Comparing with the results in each column, SVM achieved the best performance (from 91.7% to 100%) for all the target features. The lowest accuracy from SVM is 91.7% at target feature 19. The reason could be that the datasets for feature 19 contains noise and uncertainties that reduces the accuracy from all the algorithms. In that column, we can find that DT is 87.1%, KNN is 90.9, and ANN is 86.5. We compare the results, SVM (91.7) is still the best.  Figure 3 is the column chart associated with Table 5. SVM is in orange and is the highest in each column. In this article, we found a machine learning method with SVM achieved the significant accuracy (from 91.7 to 100%) to diagnose subcutaneous cyst in addressing blood flow, echo, internal echo, boundary, strong spot, and changes of parenchyma echo.

## 4. Discussion and Conclusions

In this study, a total of 132 patients from Hunan Provincial People's Hospital in China participated. Four different types of machine algorithms including decision tree (DT), support vector machine (SVM), *K*-nearest neighbors (KNN), and neural networks (NN) in machine learning method are applied for the diagnose of subcutaneous cyst by ultrasonography. Decision tree is an effective ultrasonic image classification algorithm. It can learn classification rules from unordered data [24, 25]. The decision tree algorithm uses the divide and conquer strategy to divide the search space of the problem into several subsets. From top to bottom, each node determines the next node by calculating the eigenvalue of the input sample. In the leaf node, the final classification result is given [26]. In the case of small amount of data and nondiversified eigenvalues, the construction of decision tree is simple and fast. However, if the data volume is large and the eigenvalues are large, the complexity of the decision tree algorithm will be large. Support vector machine has good performance on both small datasets and large datasets. However, with the increase of dataset size, the complexity of support vector machine also increases. At the same time, the choice of kernel function will also affect the performance of support vector machine [27–29]. *K*-nearest neighbors is a lazy and nonparametric algorithm that has the good characteristics of being simple and easy to use and has a reasonable accuracy [30].

Our research has limitations. First of all, the training set data came from the same hospital, and we did not summarize the basic information of patients and cysts. Second, no matter training or testing datasets, the sample size is relatively small. Therefore, these results need to be validated in a larger cohort to determine the value of our model in clinical practice.

All datasets are separated into two parts, which is 70% for training and 30% for testing. Results show that SVM achieved the best performance (from 91.7% to 100%) for all the target features. The machine learning method developed in this study can help doctors diagnose the ultrasonic images of patients with subcutaneous cysts more accurately. However, other prospective cohort studies should be conducted externally.

## Figures and Tables

**Figure 1:** Sample ultrasound images of subcutaneous cyst.

**Figure 2:** Workflow diagram for machine learning applied diagnosis method.

**Figure 3:** Column chart of testing results.

**Table 1:** 19 features extracted from datasets.

ID	Feature	Type
1	Gender	Categorical
2	Age	Numerical
3	None blood flow	Categorical
4	Dotted blood flow	Categorical
5	Dot-bar blood flow	Categorical
6	Rich blood flow	Categorical
7	None Echo	Categorical
8	Mixed Echo	Categorical
9	Low Echo	Categorical
10	Medium Echo	Categorical
11	High Echo	Categorical
12	Uniform internal Echo	Categorical
13	Nonuniform internal Echo	Categorical
14	Clear boundary	Categorical
15	Unclear boundary	Categorical
16	Regular form	Categorical
17	Irregular form	Categorical
18	Strong spot	Categorical
19	Changes of parenchyma Echo	Categorical

**Table 2:** Machine learning algorithms for training.

Algorithm	Accuracy (%)
Decision tree (DT)	99.2
Support vector machine (SVM)	100
*K*-nearest neighbors (KNN)	92.4
Artificial neural network (ANN)	98.5

**Table 3:** Machine learning algorithms for testing.

Algorithm	Accuracy (%)
Decision tree (DT)	96.2
Support vector machine (SVM)	100
*K*-nearest neighbors (KNN)	95.5
Artificial neural network (ANN)	98.8

**Table 4:** Testing results for target features.

Accuracy (%)	3	4	5	6	7	8	9	10
DT	96.2	97.0	98.5	93.9	98.5	97.0	95.6	98.5
SVM	100	99.2	99.2	99.2	99.2	99.2	98.8	99.2
KNN	95.5	95.5	93.9	94.7	97.0	95.5	90.2	97.0
ANN	98.8	97.7	96.2	97.0	98.5	97.7	97.7	98.5

**Table 5:** Testing results for target features.

Accuracy (%)	11	12	13	14	15	16	17	18	19
DT	98.5	95.5	95.5	96.2	98.5	97.7	97.0	85.6	87.1
SVM	99.2	100	100	100	100	100	100	92.9	91.7
KNN	98.5	96.2	96.2	97.7	97.7	90.9	90.2	87.9	90.9
ANN	97.0	99.2	98.5	99.2	99.2	99.2	99.2	83.3	86.4

## Data Availability

The labeled dataset used to support the findings of this study is available from the corresponding author upon request.
